The article "Development of improved estimators of finite population mean in simple random sampling with dual auxiliaries and its application to real world problems" was published in 2024. Journal: Heliyon.

# Development of improved estimators of finite population mean in simple random sampling with dual auxiliaries and its application to real world problems

**DOI:** 10.1016/j.heliyon.2024.e30991

**Published:** 2024-05-09

**Authors:** Khazan Sher, Muhammad Ameeq, Muhammad Muneeb Hassan, Olayan Albalawi, Ayesha Afzal

**Affiliations:** a Department of Statistics University of Peshawar, Pakistan; b Department of Statistics, The Islamia University Bahawalpur, Punjab, Pakistan; c Department of Statistics, Faculty of Science, University of Tabuk, Tabuk, Saudi Arabia; d Department of Computer Science, Air University, Islamabad, Pakistan

**Keywords:** Bias, Mean square error, Double auxiliary, Simple random sampling, Efficiency

## Abstract

In general, the incorporation of supplementary information reduces the Mean Square Error (MSE) and, consequently, enhances the precision of estimating a population parameter. This improvement relies on the appropriate application of a suitable function, with careful consideration. This study introduces two innovative families of estimators for the finite population mean, both of which exhibit superior performance in scenarios involving dual auxiliary information in simple random sampling. Expressions up to the first-order approximation, for bias, and Mean Square Error were derived, and the conditions under which these proposed families surpassed the existing estimators. Our evaluation involved the use of both real and simulated data to compute the Mean Square Error and Percent Relative Efficiency (PRE) of the estimators. A comparative analysis revealed that under the specified conditions, both proposed families yielded more precise results.

## 1 Introduction

Incorporating supplementary data alongside the primary study variable typically enhances the efficiency of the estimation techniques. Generally, the efficiency tends to improve as the number of auxiliary variables increases. The utilization of auxiliary information can significantly bolster the precision of population parameter estimators provided that an appropriate mathematical function is diligently applied. When estimating the finite population mean, various methods such as ratio, regression, and exponential estimators come into play when there is a direct correlation between the study variables and auxiliary variables. Conversely, a product estimator is employed when the correlation is negative.

Survey sampling commonly leverages supplementary data to refine estimations. This practice was first introduced by Refs. [5,11] who integrated supplementary information into ratios and regression estimation methods. Numerous authors have proposed various ratio-type estimators using auxiliary variables, including [7,8,10,14,16,17,26,28,31,41] respectively. In cases of negative correlation, alternative estimators have been introduced in the literature by Refs. [23,24,[32], [33], [34],^36^,^38^]. Additionally [2,6,9,18,21], suggested ratio-cum-product estimators for population mean. For further studies see Refs. [3,12,13,15,19,20,22,25,27,39,40,42].

Building upon the foundation work of [17,25] this study introduces two innovative families of exponential ratio-cum-product estimators. The objectives of this study are twofold.

Introducing new, precise families of population mean estimators that encompass both ratio and product estimators.

To incorporate additional population parameters such as correlation coefficients and coefficients of variation from auxiliary variables to further enhance the precision of the proposed estimator.

Hence, this study delves into the use of dual auxiliary data and evaluates the estimator's effectiveness. The remainder of the manuscript is structured as follows: Section 2 contains the methodology; existing estimators and their MSEs are discussed in Section 3; Section 4 presents the suggested estimators along with the development of bias and MSE Expressions, Section 5 details the conditions under which the proposed families outperform existing ones; and Sections 6, 7 encompass empirical and simulation studies, respectively. Section 8 presents a discussion and conclusions. The limitations are presented in Section 9, respectively.

## 2 Methodology

Let a finite population denoted as $\Omega =\left(\omega_{1},\omega_{2},\omega_{3},.....,\omega_{N}\right)$ with a total size of *N*. We aim to obtain a random sample of *n* units using the Simple Random Sampling (a sampling scheme where each unit of the population has an equal probability to enter the sample) without replacement (SRSWOR) method. Within this context, we have a study variable denoted as "*y*" and our objective is to estimate its mean. To assist in this estimation, we have access to information from two auxiliary variables, "*X”* and "*Z*" It is important to note that data pertaining to both the main study variable and the variables are readily accessible. Let $\varepsilon_{0}=\left(\bar{y}-\bar{Y}\right){\left(\bar{Y}\right)}^{-1}$, $\varepsilon_{1}=\left(\bar{x}-\bar{X}\right){\left(\bar{X}\right)}^{-1}$ and $\varepsilon_{2}=\left(\bar{z}-\bar{Z}\right){\left(\bar{Z}\right)}^{-1}$ that can satisfy the following properties.

$$E\left(\varepsilon_{0}\right)=E\left(\varepsilon_{1}\right)=E\left(\varepsilon_{2}\right)=0,E\left(\varepsilon_{0}^{2}\right)=\lambda C_{y}^{2},E\left(\varepsilon_{1}^{2}\right)=\lambda C_{x}^{2},E\left(\varepsilon_{2}^{2}\right)=\lambda C_{z}^{2},E\left(\varepsilon_{0}\varepsilon_{1}\right)=\lambda C_{yx},E\left(\varepsilon_{0}\varepsilon_{2}\right)=\lambda C_{yz}\;\text{and}\;E\left(\varepsilon_{1}\varepsilon_{2}\right)=\lambda C_{xz}\;\text{where}\;\lambda =\frac{n-N}{nN}$$

Further $\bar{Y}=N^{-1}\sum_{i=1}^{N}y_{i}$, $\bar{X}=N^{-1}\sum_{i=1}^{N}x_{i}$ and $\bar{Z}=N^{-1}\sum_{i=1}^{N}z_{i}$, $S_{y}^{2}=N^{-1}\sum_{i=1}^{N}{\left(y-\bar{Y}\right)}^{2}$, $S_{x}^{2}=N^{-1}\sum_{i=1}^{N}{\left(x-\bar{X}\right)}^{2}$, $S_{z}^{2}=N^{-1}\sum_{i=1}^{N}{\left(z-\bar{Z}\right)}^{2}$, $C_{yx}=\rho_{yx}C_{y}C_{x}$, $C_{yz}=\rho_{yz}C_{y}C_{z}$, $C_{xz}=\rho_{xz}C_{x}C_{z}$.

The integration of auxiliary information not only contributes to reducing bias but also minimizes variability in the estimation, ultimately leading to improved overall performance. Therefore, the dual auxiliary method serves as a robust means to enhance estimator efficiency by harnessing the power of additional information in the estimation process.

## 3 Estimators in literature

Numerous estimators for calculating the population mean have been developed and documented in the field of statistics. Researchers and practitioners often choose from this pool of estimators based on the specific characteristics of their data and the underlying assumptions that align with their research objectives, ensuring the most suitable and accurate estimation of the population mean.

The customary, traditional estimate of mean $EST0=\bar{y}$ is used when the data consists only a study variable. The estimator's variance is provided in Eq. (1) as

(1) $$V\left(EST0\right)={\bar{Y}}^{2}\lambda C_{y}^{2}$$

According to [29], the ratio estimator in the situation of a dual auxiliary is given in Eq. (2) as follows:

(2) $$ESTr=\bar{y}\left(\frac{\bar{X}}{\bar{x}}\right)\left(\frac{\bar{Z}}{\bar{z}}\right)$$

The *MSE* of the above ratio estimator is listed in Eq. (3) as

(3) $$MSE\left(ESTp\right)=\lambda {\bar{Y}}^{2}\left(C_{y}^{2}+C_{x}^{2}+C_{z}^{2}-2C_{yx}-2C_{yz}+2C_{xz}\right)$$

The chain ratio-product estimator proposed by [35] is given in Eq. (4) as

(4) $$ESTrp=\bar{y}\left(\frac{\bar{X}}{\bar{x}}\right)\left(\frac{\bar{z}}{\bar{Z}}\right)$$

*MSE* up to first order of approximation of the above estimator is shown in Eq. (5) as

(5) $$MSE\left(ESTrp\right)=\lambda {\bar{Y}}^{2}\left(C_{y}^{2}+C_{x}^{2}+C_{z}^{2}-2C_{yx}+2C_{yz}-2C_{xz}\right)$$

The regression estimator in dual auxiliary is given in Eq. (6) as

(6) $$ESTreg=\bar{y}+b_{1}\left(\bar{X}-\bar{x}\right)+b_{2}\left(\bar{Z}-\bar{z}\right)$$

Where $b_{1}=\frac{s_{yx}}{s_{x}^{2}}$ and $b_{2}=\frac{s_{yz}}{s_{z}^{2}}$ are the sample regression coefficient associated with $\beta_{1}=\frac{S_{yx}}{S_{x}^{2}}$ and $\beta_{2}=\frac{S_{yz}}{S_{z}^{2}}$ within the population.

The *MSE* of the regression estimator takes the following form of Eq. (7)

(7) $$MSE\left(ESTreg\right)=\lambda {\bar{Y}}^{2}C_{y}^{2}\left(1-\rho_{yx}^{2}-\rho_{yz}^{2}+2\rho_{yx}\rho_{yz}\rho_{xz}\right)$$

[21] proposed the following regression-exponential-Ratio type estimator mentioned as in Eq. (8)

(8) $$ESTs=\left[w_{1}\bar{y}-w_{2}\left(\bar{x}-\bar{X}\right)\right]\left[\alpha \left\{2-\exp\left(\frac{\bar{z}-\bar{Z}}{\bar{z}+\bar{Z}}\right)\right\}+\left(1-\alpha \right)\exp\left(\frac{\bar{Z}-\bar{z}}{\bar{z}+\bar{Z}}\right)\right]$$

Where $w_{1}$ and $w_{2}$ are minimizing constants and α takes values either 1 or 0 to have ratio exponential or product exponential estimator respectively. The ex*pre*ssion for the least *MSE* of the estimator is provided by Eq. (9).

(9) $$MSE\left(ESTs\right)≅{\bar{Y}}^{2}\left(1-\frac{\lambda C_{xz}^{2}}{4C_{x}^{2}}-\frac{\Delta_{1}^{2}}{\Delta_{2}}\right)$$

Where $\Delta_{1}=1+\left(\frac{3}{8}-\frac{\alpha }{4}\right)\lambda C_{z}^{2}-\frac{\lambda C_{yz}}{2}-\frac{\lambda C_{xz}\left(C_{xz}-C_{yx}\right)}{2C_{x}^{2}}$ and $\Delta_{2}=1+\lambda C_{y}^{2}+\left(1-\frac{\alpha }{2}\right)\lambda C_{z}^{2}-2\lambda C_{yz}-\frac{\lambda {\left(C_{xz}-C_{yx}\right)}^{2}}{C_{x}^{2}}$.

The proposed estimator by [12] in two auxiliary takes the exponential form listed in Eq. (10) as follow

(10) $$ESTh=\left\{w_{3}\bar{y}+w_{4}\left(\frac{\bar{X}-\bar{x}}{\bar{X}}\right)+w_{5}\left(\frac{\bar{Z}-\bar{z}}{\bar{Z}}\right)\right\}\exp\left[\frac{u\left(\bar{X}-\bar{x}\right)}{u\left(\bar{X}+\bar{x}\right)+2v}\right]$$

Where $w_{3}$, $w_{4}$ and $w_{5}$ are the minimizing constants the values of whom are to be obtained so that the resulting *MSE* is minimum. where u and v are generalizing constants, whose values consists of different parameters of the auxiliary variables. Let $\eta =\frac{u\bar{X}}{u\bar{X}+v}$ then minimum *MSE* of estimator is listed Eq. (11) as

(11) $$MSE\left(ESTh\right)≅{\bar{Y}}^{2}\lambda C_{y}^{2}\left(1-\rho_{yx}^{2}\right)-H_{1}-H_{2}$$

Where $H_{1}=\frac{{\bar{Y}}^{2}{\left(\eta^{2}C_{x}^{4}-8C_{yx}^{2}+8C_{y}^{2}C_{x}^{2}\right)}^{2}}{64C_{x}^{4}\left\{1+C_{y}^{2}\left(1-\rho_{yx}^{2}\right)\right\}}$ and $H_{2}=\frac{{\bar{Y}}^{2}{\left(\eta^{2}C_{x}^{2}-8\right)}^{2}{\left(C_{x}^{2}C_{yz}-C_{yx}C_{xz}\right)}^{2}}{64C_{x}^{4}C_{z}^{2}\left(1-\rho_{xz}^{2}\right)\left\{1+C_{y}^{2}\left(1-\rho_{yx}^{2}\right)\right\}\left\{1+C_{y}^{2}\left(1-\rho_{y.xz}^{2}\right)\right\}}$.

[30] Proposed the following product estimator in Eq. (12)

(12) $$ESTsn=w_{6}\bar{y}+w_{7}\bar{y}{\left(\frac{\bar{x}}{\bar{X}}\right)}^{\alpha_{1}}+w_{8}\bar{y}{\left(\frac{\bar{z}}{\bar{Z}}\right)}^{\alpha_{2}}$$

Here the $w_{6}$, $w_{7}$ and $w_{8}$ are the minimizing constants values of whom are obtained so that the *MSE* is least, $\alpha_{1}$ and $\alpha_{2}$ can take any value either negative or positive. For $w_{6}=\frac{\Psi_{0}}{\Psi }$, $w_{7}=\frac{\Psi_{1}}{\Psi }$, and $w_{8}=\frac{\Psi_{2}}{\Psi }$ the minimum *MSE* of the Singh and Nigam's estimator is provided in Eq. (13) as

(13) $$MSE\left(ESTsn\right)≅{\bar{Y}}^{2}\left[1-\frac{\Psi_{0}+A_{6}\Psi_{1}+A_{7}\Psi_{2}}{\Psi }\right]$$

Where $\Psi =A_{0}\left(A_{1}A_{2}-A_{5}^{2}\right)-A_{3}\left(A_{2}A_{3}-A_{4}A_{5}\right)+A_{4}\left(A_{3}A_{5}-A_{1}A_{4}\right)$, $\Psi_{0}=\left(A_{1}A_{2}-A_{5}^{2}\right)-A_{3}\left(A_{2}A_{6}-A_{5}A_{7}\right)+A_{4}\left(A_{5}A_{6}-A_{1}A_{7}\right)\Psi_{1}=A_{0}\left(A_{2}A_{6}-A_{5}A_{7}\right)-\left(A_{2}A_{3}-A_{4}A_{5}\right)+A_{4}\left(A_{3}A_{7}-A_{4}A_{6}\right)$ and $\Psi_{2}=A_{0}\left(A_{1}A_{7}-A_{5}A_{6}\right)-A_{3}\left(A_{3}A_{7}-A_{4}A_{6}\right)+\left(A_{3}A_{5}-A_{1}A_{4}\right)$.

Further $A_{0}=1+\lambda C_{y}^{2}$, $A_{1}=1+\lambda \left\{C_{y}^{2}+4\alpha_{1}C_{yx}+\alpha_{1}\left(2\alpha_{1}-1\right)C_{x}^{2}\right\}$, $A_{2}=1+\lambda \left\{C_{y}^{2}+4\alpha_{2}C_{yz}+\alpha_{2}\left(2\alpha_{2}-1\right)C_{z}^{2}\right\}A_{3}=1+\lambda \left\{C_{y}^{2}+2\alpha_{1}C_{yx}+\frac{\alpha_{1}\left(\alpha_{1}-1\right)}{2}C_{x}^{2}\right\}$, $A_{4}=1+\lambda \left\{C_{y}^{2}+2\alpha_{2}C_{yz}+\frac{\alpha_{2}\left(\alpha_{2}-1\right)}{2}C_{z}^{2}\right\}$, $A_{5}=1+\lambda \left\{C_{y}^{2}+2\alpha_{1}C_{yx}+2\alpha_{2}C_{yz}+\alpha_{1}\alpha_{2}C_{xz}+\frac{\alpha_{1}\left(\alpha_{1}-1\right)}{2}C_{x}^{2}+\frac{\alpha_{2}\left(\alpha_{2}-1\right)}{2}C_{z}^{2}\right\}$.

$$A_{6}=1+\frac{\lambda \alpha_{1}}{2}\left(\alpha_{1}+2C_{yx}{\left(C_{x}^{2}\right)}^{-1}-1\right)C_{x}^{2}\;\text{and}\;A_{7}=1+\frac{\lambda \alpha_{2}}{2}\left(\alpha_{2}+2C_{yz}{\left(C_{z}^{2}\right)}^{-1}-1\right)C_{z}^{2}$$

## 4 Proposed estimator

This segment *Pre*sents two families of suggested estimators for the finite population mean through the utilization of double secondary variables within the framework of simple random sampling. Furthermore, within this segment, we derive ex*pre*ssions for both bias and *MSE*.

### 4.1 First proposed estimator

[25] proposed exponential ratio-cum-product estimator in single auxiliary case which gives efficient results even if the correlation between the variables is not strong enough.

$$T_{Shb}=\left[\varphi_{1}\bar{y}+\varphi_{2}\right]\exp\left[\frac{u\left(\bar{X}-\bar{x}\right)}{u\left(\bar{X}+\bar{x}\right)+2v}\right]$$

Here $\varphi_{1}$ and $\varphi_{2}$ are constants whose values are to be determined so that the resultant MSE is minimum, *u* and *v* are generalizing constants which can adopt any value from the known values of the parameters of the supplementary variable. [21] Introduced the below estimator in the presence of two auxiliary variables.

$$T_{SA}=\left[\varphi_{3}\bar{y}+\varphi_{4}\left(\bar{x}-\bar{X}\right)\right]\left[\alpha \left\{2-\exp\left[\frac{\bar{z}-\bar{Z}}{\bar{Z}+\bar{z}}\right]\right\}+\left(1-\alpha \right)exp\left[\frac{\bar{Z}-\bar{z}}{\bar{Z}+\bar{z}}\right]\right]$$

Again in this estimator the $\varphi_{3}$ and $\varphi_{4}$ are minimizing constants whose values are obtained by the differentiating the MSE expression and α can take value either 0 or 1.

Motivated from these works a novel family of estimators for population mean is suggested in Eq. (14) below by modifying [21].

(14) $$ESTp1=\left[t_{1}\bar{y}+t_{2}\right]\left[l\frac{\bar{X}}{\bar{x}}\left\{2-\exp\left[\frac{u\left(\bar{z}-\bar{Z}\right)}{u\left(\bar{Z}+\bar{z}\right)+2v}\right]\right\}+\left(1-l\right)\frac{\bar{x}}{\bar{X}}\exp\left[\frac{u\left(\bar{Z}-\bar{z}\right)}{u\left(\bar{Z}+\bar{z}\right)+2v}\right]\right]$$

Several estimators can be produced from the above estimator by substituting different values of u, v and l. here $t_{1}$ and $t_{2}$ are the minimizing constants whose values are determined by minimizing the *MSE* and u, v and l are the generalizing constants which can assume any suitable value or any known parameter of the population. For obtaining the *MSE* of the estimator, we can ex*pre*ss the above Eq. (14) in terms of sampling errors as below

(15) $$ESTp1=\left[t_{1}\bar{Y}\left(1+\varepsilon_{0}\right)+t_{2}\right]\left[\begin{array}{c} l\frac{\bar{X}}{\bar{X}\left(1+\varepsilon_{1}\right)}\left\{2-\exp\left[\frac{u\left(\bar{Z}\left(1+\varepsilon_{2}\right)-\bar{Z}\right)}{u\left(\bar{Z}+\bar{Z}\left(1+\varepsilon_{2}\right)\right)+2v}\right]\right\}\\ +\left(1-l\right)\frac{\bar{X}\left(1+\varepsilon_{1}\right)}{\bar{X}}\exp\left[\frac{u\left(\bar{Z}-\bar{Z}\left(1+\varepsilon_{2}\right)\right)}{u\left(\bar{Z}+\bar{Z}\left(1+\varepsilon_{2}\right)\right)+2v}\right] \end{array}\right]$$

Simplifying Eq. (15) by applying Taylor series the following equation is obtained in terms of sampling errors

(16) $$ESTp1≃t_{1}\bar{Y}\left(1+\varepsilon_{0}+\vartheta_{1}\varepsilon_{1}+\vartheta_{1}\varepsilon_{0}\varepsilon_{1}-\vartheta_{2}\varepsilon_{2}-\vartheta_{2}\varepsilon_{0}\varepsilon_{2}+l\varepsilon_{1}^{2}+\vartheta_{3}\varepsilon_{1}\varepsilon_{2}+\vartheta_{4}\varepsilon_{2}^{2}\right)+t_{2}\left(1+\vartheta_{1}\varepsilon_{1}-\vartheta_{2}\varepsilon_{2}+l\varepsilon_{1}^{2}+\vartheta_{3}\varepsilon_{1}\varepsilon_{2}+\vartheta_{4}\varepsilon_{2}^{2}\right)$$

Where $\vartheta_{1}=1-2l$, $\vartheta_{2}=\frac{\tau }{2}$, $\vartheta_{3}=\left(l-\frac{1}{2}\right)\tau$, $\vartheta_{4}=\frac{1}{8}\left(3-2l\right)\tau^{2}$ and $\tau =\frac{u\bar{Z}}{u\bar{Z}+v}$.

Now the ex*pre*ssion mentioned below is obtained by subtracting $\bar{Y}$ from each side of Eq. (16)

(17) $$ESTp1-\bar{Y}=t_{1}\bar{Y}\left(1+\varepsilon_{0}+\vartheta_{1}\varepsilon_{1}+\vartheta_{1}\varepsilon_{0}\varepsilon_{1}-\vartheta_{2}\varepsilon_{2}-\vartheta_{2}\varepsilon_{0}\varepsilon_{2}+l\varepsilon_{1}^{2}+\vartheta_{3}\varepsilon_{1}\varepsilon_{2}+\vartheta_{4}\varepsilon_{2}^{2}\right)+t_{2}\left(1+\vartheta_{1}\varepsilon_{1}-\vartheta_{2}\varepsilon_{2}+l\varepsilon_{1}^{2}+\vartheta_{3}\varepsilon_{1}\varepsilon_{2}+\vartheta_{4}\varepsilon_{2}^{2}\right)-\bar{Y}$$

After taking expectation on Eq. (17) the following bias ex*pre*ssion is obtained as in Eq. (18)

(18) $$Bias\left(ESTp1\right)≃t_{1}\bar{Y}\left(1+\vartheta_{1}\lambda C_{yx}-\vartheta_{2}\lambda C_{yz}\varepsilon_{2}+l\lambda C_{x}^{2}+\vartheta_{3}\lambda C_{xz}+\vartheta_{4}\lambda C_{z}^{2}\right)+t_{2}\left(1+l\lambda C_{x}^{2}+\vartheta_{3}\lambda C_{xz}+\vartheta_{4}\lambda C_{z}^{2}\right)-\bar{Y}$$

Let's take square and expectation on Eq. (17) to have an ex*pre*ssion for *MSE*

$$E{\left(ESTp1-\bar{Y}\right)}^{2}≃E\left[\begin{array}{c} t_{1}^{2}{\bar{Y}}^{2}\left\{1+\varepsilon_{0}^{2}+\left(\vartheta_{1}^{2}+2l\right)\varepsilon_{1}^{2}+\left(\vartheta_{2}^{2}+2\vartheta_{4}\right)\varepsilon_{2}^{2}+4\vartheta_{1}\varepsilon_{0}\varepsilon_{1}-4\vartheta_{2}\varepsilon_{0}\varepsilon_{2}+2\left(\vartheta_{3}-\vartheta_{1}\vartheta_{2}\right)\varepsilon_{1}\varepsilon_{2}\right\}\\ +t_{2}^{2}\left\{1+\left(\vartheta_{1}^{2}+2l\right)\varepsilon_{1}^{2}+\left(\vartheta_{2}^{2}+2\vartheta_{4}\right)\varepsilon_{2}^{2}+2\left(\vartheta_{3}-\vartheta_{1}\vartheta_{2}\right)\varepsilon_{1}\varepsilon_{2}\right\}+{\bar{Y}}^{2}\\ -2t_{1}{\bar{Y}}^{2}\left(1+l\varepsilon_{1}^{2}+\vartheta_{4}\varepsilon_{2}^{2}+\vartheta_{1}\varepsilon_{0}\varepsilon_{1}-\vartheta_{2}\varepsilon_{0}\varepsilon_{2}+\vartheta_{3}\varepsilon_{1}\varepsilon_{2}\right)-2t_{2}\bar{Y}\left(1+l\varepsilon_{1}^{2}+\vartheta_{4}\varepsilon_{2}^{2}+\vartheta_{3}\varepsilon_{1}\varepsilon_{2}\right)\\ +2t_{1}t_{2}\bar{Y}\left\{1+\left(\vartheta_{1}^{2}+2l\right)\varepsilon_{1}^{2}+\left(\vartheta_{2}^{2}+2\vartheta_{4}\right)\varepsilon_{2}^{2}+2\vartheta_{1}\varepsilon_{0}\varepsilon_{1}-2\vartheta_{2}\varepsilon_{0}\varepsilon_{2}+2\left(\vartheta_{3}-\vartheta_{1}\vartheta_{2}\right)\varepsilon_{1}\varepsilon_{2}\right\} \end{array}\right]$$

Or the above equation can be written in Eq. (19) as

(19) $$MSE\left(ESTp1\right)≃t_{1}^{2}{\bar{Y}}^{2}\left\{1+\lambda C_{y}^{2}+\left(\vartheta_{1}^{2}+2l\right)\lambda C_{x}^{2}+\left(\vartheta_{2}^{2}+2\vartheta_{4}\right)\lambda C_{z}^{2}+4\vartheta_{1}\lambda C_{yx}-4\vartheta_{2}\lambda C_{yz}+2\left(\vartheta_{3}-\vartheta_{1}\vartheta_{2}\right)\lambda C_{xz}\right\}+t_{2}^{2}\left\{1+\left(\vartheta_{1}^{2}+2l\right)\lambda C_{x}^{2}+\left(\vartheta_{2}^{2}+2\vartheta_{4}\right)\lambda C_{z}^{2}+2\left(\vartheta_{3}-\vartheta_{1}\vartheta_{2}\right)\lambda C_{xz}\right\}+{\bar{Y}}^{2}-2t_{1}{\bar{Y}}^{2}\left(1+l\lambda C_{x}^{2}+\vartheta_{4}\lambda C_{z}^{2}+\vartheta_{1}\lambda C_{yx}-\vartheta_{2}\lambda C_{yz}+\vartheta_{3}\lambda C_{xz}\right)-2t_{2}\bar{Y}\left(1+l\lambda C_{x}^{2}+\vartheta_{4}\lambda C_{z}^{2}+\vartheta_{3}\lambda C_{xz}\right)+2t_{1}t_{2}\bar{Y}\left\{1+\left(\vartheta_{1}^{2}+2l\right)\lambda C_{x}^{2}+\left(\vartheta_{2}^{2}+2\vartheta_{4}\right)\lambda C_{z}^{2}+2\vartheta_{1}\lambda C_{yx}-2\vartheta_{2}\lambda C_{yz}+2\left(\vartheta_{3}-\vartheta_{1}\vartheta_{2}\right)\lambda C_{xz}\right\}$$

The simplified form of the above equation is provided in Eq. (20) as follow

(20) $$MSE\left(ESTp1\right)≃t_{1}^{2}{\bar{Y}}^{2}A_{\mathrm{pr}}+t_{2}^{2}B_{\mathrm{pr}}+{\bar{Y}}^{2}-2t_{1}{\bar{Y}}^{2}C_{\mathrm{pr}}-2t_{2}\bar{Y}D_{\mathrm{pr}}+2t_{1}t_{2}\bar{Y}E_{\mathrm{pr}}$$

Where $A_{\mathrm{pr}}=1+\lambda C_{y}^{2}+\left(\vartheta_{1}^{2}+2l\right)\lambda C_{x}^{2}+\left(\vartheta_{2}^{2}+2\vartheta_{4}\right)\lambda C_{z}^{2}+4\vartheta_{1}\lambda C_{yx}-4\vartheta_{2}\lambda C_{yz}+2\left(\vartheta_{3}-\vartheta_{1}\vartheta_{2}\right)\lambda C_{xz}$, $B_{\mathrm{pr}}=1+\left(\vartheta_{1}^{2}+2l\right)\lambda C_{x}^{2}+\left(\vartheta_{2}^{2}+2\vartheta_{4}\right)\lambda C_{z}^{2}+2\left(\vartheta_{3}-\vartheta_{1}\vartheta_{2}\right)\lambda C_{xz}$, $C_{\mathrm{pr}}=1+l\lambda C_{x}^{2}+\vartheta_{4}\lambda C_{z}^{2}+\vartheta_{1}\lambda C_{yx}-\vartheta_{2}\lambda C_{yz}+\vartheta_{3}\lambda C_{xz}$, $D_{\mathrm{pr}}=1+l\lambda C_{x}^{2}+\vartheta_{4}\lambda C_{z}^{2}+\vartheta_{3}\lambda C_{xz}$ and $E_{\mathrm{pr}}=1+\left(\vartheta_{1}^{2}+2l\right)\lambda C_{x}^{2}+\left(\vartheta_{2}^{2}+2\vartheta_{4}\right)\lambda C_{z}^{2}+2\vartheta_{1}\lambda C_{yx}-2\vartheta_{2}\lambda C_{yz}+2\left(\vartheta_{3}-\vartheta_{1}\vartheta_{2}\right)\lambda C_{xz}$.

Applying mathematical rule to obtain the optimum values of *t*_*1*_ and *t*_*2*_ from Eq. (20) as follow

(21) $$\frac{\partial MSE\left(ESTp1\right)}{\partial t_{1}}=0\Rightarrow t_{1}{\bar{Y}}^{2}A_{\mathrm{pr}}+t_{2}\bar{Y}E_{\mathrm{pr}}-{\bar{Y}}^{2}C_{\mathrm{pr}}=0$$

(22) $$\frac{\partial MSE\left(ESTp1\right)}{\partial t_{2}}=0\Rightarrow t_{1}\bar{Y}E_{\mathrm{pr}}+t_{2}B_{\mathrm{pr}}-\bar{Y}D_{\mathrm{pr}}=0$$

Solving Eq. (21) and Eq. (22) simultaneously the following values of *t*_*1*_ and *t*_*2*_ are obtained.

$t_{1}=\frac{B_{\mathrm{pr}}C_{\mathrm{pr}}-D_{\mathrm{pr}}E_{\mathrm{pr}}}{A_{\mathrm{pr}}B_{\mathrm{pr}}-E_{\mathrm{pr}}^{2}}$ and $t_{2}=\frac{\bar{Y}\left(A_{\mathrm{pr}}D_{\mathrm{pr}}-C_{\mathrm{pr}}E_{\mathrm{pr}}\right)}{A_{\mathrm{pr}}B_{\mathrm{pr}}-E_{\mathrm{pr}}^{2}}$.with these values the minimum *MSE* of the estimator adopts the following form

(23) $$MSE{\left(ESTp1\right)}_{\min}={\bar{Y}}^{2}\left[1-\frac{A_{\mathrm{pr}}D_{\mathrm{pr}}^{2}+B_{\mathrm{pr}}C_{\mathrm{pr}}^{2}-2C_{\mathrm{pr}}D_{\mathrm{pr}}E_{\mathrm{pr}}}{A_{\mathrm{pr}}B_{\mathrm{pr}}-E_{\mathrm{pr}}^{2}}\right]$$

This *MSE* Eq. (23) is supposed to be minimum relative to the other competing estimators for finite population mean for different values of *u, v* and *ℓ.*

### 4.2 Second proposed estimator

A ratio cum product estimator was introduced by [4] for the finite population mean in the existence of one supplementary variable.

$$T_{CS}=\bar{y}\left[\alpha \frac{\bar{X}}{\bar{x}}+\left(1-\alpha \right)\frac{\bar{x}}{\bar{X}}\right]$$

Modifying by [4] incorporating the idea of [25] and using the dual auxiliaries a novel and effective modified exponential estimator is produced as.

(24) $$ESTp2=\left[t_{3}\bar{y}+t_{4}\right]\left[l\frac{\bar{X}}{\bar{x}}+\left(1-l\right)\frac{\bar{x}}{\bar{X}}\right]\exp\left[\frac{u\left(\bar{Z}-\bar{z}\right)}{u\left(\bar{z}+\bar{Z}\right)+2v}\right]$$

Where in Eq. (24) t_3_ and t_4_ are the minimizing constants and ℓ, *u* and *v* are the same as defined in section 4.1. The following different forms of estimators are obtained by putting different values of the l, u and v.

Table 1 shows some of the all estimators that can be deduced from the proposed families of the estimators. To find the *MSE* of the *ESTp2* estimator we ex*pre*ss Eq. (24) in terms of sampling errors as follows

(25) $$ESTp2=\left[t_{3}\bar{Y}\left(1+\varepsilon_{0}\right)+t_{4}\right]\left[l{\left(1+\varepsilon_{1}\right)}^{-1}+\left(1-l\right)\left(1+\varepsilon_{1}\right)\right]\exp\left[\frac{u\left(\bar{Z}-\bar{Z}\left(1+\varepsilon_{2}\right)\right)}{u\left(\bar{Z}\left(1+\varepsilon_{2}\right)+\bar{Z}\right)+2v}\right]$$

**Table 1:** Different estimators deduced from *ESTp1* and *ESTp2*.

S.No	u	v	l	Estimators from *ESTp1*	Estimators from *ESTp2*
1	1	0	1	$ESTp1=\left[t_{1}\bar{y}+t_{2}\right]\left[\frac{\bar{X}}{\bar{x}}\right]\left\{2-\exp\left[\frac{\bar{z}-\bar{Z}}{\bar{Z}+\bar{z}}\right]\right\}$	$ESTp2=\left[t_{3}\bar{y}+t_{4}\right]\left[\frac{\bar{X}}{\bar{x}}\right]\exp\left[\frac{\bar{Z}-\bar{z}}{\bar{Z}+\bar{z}}\right]$
2	$\rho_{yz}$	1	1	$ESTp1=\left[t_{1}\bar{y}+t_{2}\right]\left[\frac{\bar{X}}{\bar{x}}\right]\left\{2-\exp\left[\frac{\rho_{yz}\left(\bar{z}-\bar{Z}\right)}{\rho_{yz}\left(\bar{Z}+\bar{z}\right)+2}\right]\right\}$	$ESTp2=\left[t_{3}\bar{y}+t_{4}\right]\left[\frac{\bar{X}}{\bar{x}}\right]\exp\left[\frac{\rho_{yz}\left(\bar{Z}-\bar{z}\right)}{\rho_{yz}\left(\bar{Z}+\bar{z}\right)+2}\right]$
3	1	$C_{z}$	1	$ESTp1=\left[t_{1}\bar{y}+t_{2}\right]\left[\frac{\bar{X}}{\bar{x}}\right]\left\{2-\exp\left[\frac{\left(\bar{z}-\bar{Z}\right)}{\left(\bar{Z}+\bar{z}\right)+2C_{z}}\right]\right\}$	$ESTp2=\left[t_{3}\bar{y}+t_{4}\right]\left[\frac{\bar{X}}{\bar{x}}\right]\exp\left[\frac{\left(\bar{Z}-\bar{z}\right)}{\left(\bar{Z}+\bar{z}\right)+2C_{z}}\right]$
4	1	0	0	$ESTp1=\left[t_{1}\bar{y}+t_{2}\right]\left[\frac{\bar{x}}{\bar{X}}\right]\exp\left[\frac{\bar{Z}-\bar{z}}{\bar{Z}+\bar{z}}\right]$	$ESTp2=\left[t_{3}\bar{y}+t_{4}\right]\left[\frac{\bar{x}}{\bar{X}}\right]\exp\left[\frac{\bar{Z}-\bar{z}}{\bar{Z}+\bar{z}}\right]$
5	$\rho_{yz}$	1	0	$ESTp1=\left[t_{1}\bar{y}+t_{2}\right]\left[\frac{\bar{x}}{\bar{X}}\right]\exp\left[\frac{\rho_{yz}\left(\bar{Z}-\bar{z}\right)}{\rho_{yz}\left(\bar{Z}+\bar{z}\right)+2}\right]$	$ESTp2=\left[t_{3}\bar{y}+t_{4}\right]\left[\frac{\bar{x}}{\bar{X}}\right]\exp\left[\frac{\rho_{yz}\left(\bar{Z}-\bar{z}\right)}{\rho_{yz}\left(\bar{Z}+\bar{z}\right)+2}\right]$
6	1	$C_{z}$	0	$ESTp1=\left[t_{1}\bar{y}+t_{2}\right]\left[\frac{\bar{x}}{\bar{X}}\right]\exp\left[\frac{\left(\bar{Z}-\bar{z}\right)}{\left(\bar{Z}+\bar{z}\right)+2C_{z}}\right]$	$ESTp2=\left[t_{3}\bar{y}+t_{4}\right]\left[\frac{\bar{x}}{\bar{X}}\right]\exp\left[\frac{\left(\bar{Z}-\bar{z}\right)}{\left(\bar{Z}+\bar{z}\right)+2C_{z}}\right]$
7	1	0	$\frac{1}{2}$	$ESTp1=\left[t_{1}\bar{y}+t_{2}\right]\frac{1}{2}\left[\frac{\bar{X}}{\bar{x}}\left\{2-\exp\left[\frac{\bar{z}-\bar{Z}}{\bar{Z}+\bar{z}}\right]\right\}+\frac{\bar{x}}{\bar{X}}\exp\left[\frac{\bar{Z}-\bar{z}}{\bar{Z}+\bar{z}}\right]\right]$	$ESTp2=\left[t_{3}\bar{y}+t_{4}\right]\left[\frac{1}{2}\left\{\frac{\bar{X}}{\bar{x}}+\frac{\bar{x}}{\bar{X}}\right\}\right]\exp\left[\frac{\bar{Z}-\bar{z}}{\bar{Z}+\bar{z}}\right]$
8	1	1	$\frac{1}{2}$	$ESTp1=\left[t_{1}\bar{y}+t_{2}\right]\frac{1}{2}\left[\frac{\bar{X}}{\bar{x}}\left\{2-\exp\left[\frac{\bar{z}-\bar{Z}}{\left(\bar{Z}+\bar{z}\right)+2}\right]\right\}+\frac{\bar{x}}{\bar{X}}\exp\left[\frac{\bar{Z}-\bar{z}}{\left(\bar{Z}+\bar{z}\right)+2}\right]\right]$	$ESTp2=\left[t_{3}\bar{y}+t_{4}\right]\left[\frac{1}{2}\left\{\frac{\bar{X}}{\bar{x}}+\frac{\bar{x}}{\bar{X}}\right\}\right]\exp\left[\frac{\bar{Z}-\bar{z}}{\left(\bar{Z}+\bar{z}\right)+2}\right]$
9	1	$C_{z}$	$\frac{1}{2}$	$ESTp1=\left[t_{1}\bar{y}+t_{2}\right]\frac{1}{2}\left[\frac{\bar{X}}{\bar{x}}\left\{2-\exp\left[\frac{\left(\bar{z}-\bar{Z}\right)}{\left(\bar{Z}+\bar{z}\right)+2C_{z}}\right]\right\}+\frac{\bar{x}}{\bar{X}}\exp\left[\frac{\left(\bar{Z}-\bar{z}\right)}{\left(\bar{Z}+\bar{z}\right)+2C_{z}}\right]\right]$	$ESTp2=\left[t_{3}\bar{y}+t_{4}\right]\left[\frac{1}{2}\left\{\frac{\bar{X}}{\bar{x}}+\frac{\bar{x}}{\bar{X}}\right\}\right]\exp\left[\frac{\left(\bar{Z}-\bar{z}\right)}{\left(\bar{Z}+\bar{z}\right)+2C_{z}}\right]$
10	$\rho_{yz}$	$C_{z}$	$\frac{1}{2}$	$ESTp1=\left[t_{1}\bar{y}+t_{2}\right]\frac{1}{2}\left[\frac{\bar{X}}{\bar{x}}\left\{2-\exp\left[\frac{\rho_{yz}\left(\bar{z}-\bar{Z}\right)}{\rho_{yz}\left(\bar{Z}+\bar{z}\right)+2C_{z}}\right]\right\}+\frac{\bar{x}}{\bar{X}}\exp\left[\frac{\rho_{yz}\left(\bar{Z}-\bar{z}\right)}{\rho_{yz}\left(\bar{Z}+\bar{z}\right)+2C_{z}}\right]\right]$	$ESTp2=\left[t_{3}\bar{y}+t_{4}\right]\left[\frac{1}{2}\left\{\frac{\bar{X}}{\bar{x}}+\frac{\bar{x}}{\bar{X}}\right\}\right]\exp\left[\frac{\rho_{yz}\left(\bar{Z}-\bar{z}\right)}{\rho_{yz}\left(\bar{Z}+\bar{z}\right)+2C_{z}}\right]$

After simplifying Eq. (25) the difference equation is given by

(26) $$ESTp2-\bar{Y}=\left(t_{3}-1\right)\bar{Y}+k_{3}\bar{Y}\left(w_{1}\varepsilon_{1}+l\varepsilon_{1}^{2}-w_{2}\varepsilon_{2}+w_{3}\varepsilon_{2}^{2}-w_{4}\varepsilon_{1}\varepsilon_{2}\right)+t_{4}\left(1+w_{1}\varepsilon_{1}+l\varepsilon_{1}^{2}-w_{2}\varepsilon_{2}+w_{3}\varepsilon_{2}^{2}-w_{4}\varepsilon_{1}\varepsilon_{2}\right)+t_{3}\bar{Y}\left(\varepsilon_{0}+w_{1}\varepsilon_{0}\varepsilon_{1}-w_{2}\varepsilon_{0}\varepsilon_{2}\right)$$

Where $w_{1}=1-2l$, $w_{2}=\frac{1}{2}\tau$, $w_{3}=\frac{3}{8}\tau^{2}$ and $w_{4}=\frac{1}{2}\tau \left(1-2l\right)$.

The Bias of the estimator up to first order of approximation by taking the expectation of Eq. (26) is given in Eq. (27) as

(27) $$Bias\left(ESTp2\right)≃\left(t_{3}-1\right)\bar{Y}+t_{3}\bar{Y}\lambda \left(lC_{x}^{2}+w_{3}C_{z}^{2}-w_{4}C_{xz}\right)+k_{1}\bar{Y}\lambda \left(w_{1}C_{yx}-w_{2}C_{yz}\right)+k_{2}\left(1+l\lambda C_{x}^{2}+w_{3}\lambda C_{z}^{2}-w_{4}\lambda C_{xz}\right)$$

Taking square of Eq. (26) and applying expectation we have

$$E{\left(ESTp2-\bar{Y}\right)}^{2}≃E\left[\begin{array}{c} {\left(k_{1}-1\right)}^{2}{\bar{Y}}^{2}+k_{1}^{2}{\bar{Y}}^{2}\left\{\varepsilon_{0}^{2}+\left(w_{1}^{2}+2l\right)\varepsilon_{1}^{2}+\left(w_{2}^{2}+2w_{3}\right)\varepsilon_{2}^{2}-2\left(w_{4}+w_{1}w_{2}\right)\varepsilon_{1}\varepsilon_{2}+4w_{1}\varepsilon_{0}\varepsilon_{1}-4w_{2}\varepsilon_{0}\varepsilon_{2}\right\}\\ +k_{2}^{2}\left\{1+\left(w_{1}^{2}+2l\right)\varepsilon_{1}^{2}+\left(w_{2}^{2}+2w_{3}\right)\varepsilon_{2}^{2}-2\left(w_{4}+w_{1}w_{2}\right)\varepsilon_{1}\varepsilon_{2}\right\}\\ -2k_{1}{\bar{Y}}^{2}\left(l\varepsilon_{1}^{2}+w_{3}\varepsilon_{2}^{2}-w_{4}\varepsilon_{1}\varepsilon_{2}+w_{1}\varepsilon_{0}\varepsilon_{1}-w_{2}\varepsilon_{0}\varepsilon_{2}\right)-2k_{2}\bar{Y}\left(1+l\varepsilon_{1}^{2}+w_{3}\varepsilon_{2}^{2}-w_{4}\varepsilon_{1}\varepsilon_{2}\right)\\ +2k_{1}k_{2}\bar{Y}\left\{1+\left(w_{1}^{2}+2l\right)\varepsilon_{1}^{2}+\left(w_{2}^{2}+2w_{3}\right)\varepsilon_{2}^{2}-2\left(w_{4}+w_{1}w_{2}\right)\varepsilon_{1}\varepsilon_{2}+2w_{1}\varepsilon_{0}\varepsilon_{1}-2w_{2}\varepsilon_{0}\varepsilon_{2}\right\} \end{array}\right]$$

or

(28) $$MSE\left(ESTp2\right)≅{\left(t_{3}-1\right)}^{2}{\bar{Y}}^{2}+t_{3}^{2}{\bar{Y}}^{2}\left\{\begin{array}{c} \lambda C_{y}^{2}+\left(w_{1}^{2}+2l\right)\lambda C_{x}^{2}+\left(w_{2}^{2}+2w_{3}\right)\lambda C_{z}^{2}\\ -2\left(w_{4}+w_{1}w_{2}\right)\lambda C_{xz}+4w_{1}\lambda C_{yx}-4w_{2}\lambda C_{yz} \end{array}\right\}+t_{4}^{2}\left\{1+\left(w_{1}^{2}+2l\right)\lambda C_{x}^{2}+\left(w_{2}^{2}+2w_{3}\right)\lambda C_{z}^{2}-2\left(w_{4}+w_{1}w_{2}\right)\lambda C_{xz}\right\}-2t_{3}{\bar{Y}}^{2}\left(l\lambda C_{x}^{2}+w_{3}\lambda C_{z}^{2}-w_{4}\lambda C_{xz}+w_{1}\lambda C_{yx}-w_{2}\lambda C_{yz}\right)-2t_{4}\bar{Y}\left(1+l\lambda C_{x}^{2}+w_{3}\lambda C_{z}^{2}-w_{4}\lambda C_{xz}\right)+2t_{3}t_{4}\bar{Y}\left\{\begin{array}{c} 1+\left(w_{1}^{2}+2l\right)\lambda C_{x}^{2}+\left(w_{2}^{2}+2w_{3}\right)\lambda C_{z}^{2}\\ -2\left(w_{4}+w_{1}w_{2}\right)\lambda C_{xz}+2w_{1}\lambda C_{yx}-2w_{2}\lambda C_{yz} \end{array}\right\}$$

Applying mathematical rules on Eq. (28) to find the optimum values of *t*_*3*_ and *t*_*4*_ as follow

(29) $$\frac{\partial MSE\left(ESTp2\right)}{\partial t_{3}}=0\Rightarrow 2\left(t_{3}-1\right){\bar{Y}}^{2}+2t_{3}{\bar{Y}}^{2}A_{p2}-2{\bar{Y}}^{2}D_{p2}+2t_{4}\bar{Y}E_{p2}=0$$

and

(30) $$\frac{\partial MSE\left(ESTp2\right)}{\partial t_{4}}=0\Rightarrow 2t_{4}B_{p2}-2\bar{Y}D_{p2}+2t_{3}\bar{Y}E_{p2}=0$$

Solving both the equations Eq. (29) and Eq. (30) simultaneously, we have

$$t_{3}=\frac{B_{p2}C_{p2}-D_{p2}E_{p2}+B_{p2}}{A_{p2}B_{p2}-E_{p2}^{2}+B_{p2}}\;\text{and}\;t_{4}=\frac{\bar{Y}\left(A_{p2}D_{p2}-C_{p2}E_{p2}+D_{p2}-E_{p2}\right)}{A_{p2}B_{p2}-E_{p2}^{2}+B_{p2}}$$

Where $A_{p2}=\lambda \left\{C_{y}^{2}+\left(w_{1}^{2}+2l\right)C_{x}^{2}+\left(w_{2}^{2}+2w_{3}\right)C_{z}^{2}-2\left(w_{4}+w_{1}w_{2}\right)C_{xz}+4w_{1}C_{yx}-4w_{2}C_{yz}\right\}$.

$$B_{p2}=1+\lambda \left\{\left(w_{1}^{2}+2l\right)C_{x}^{2}+\left(w_{2}^{2}+2w_{3}\right)C_{z}^{2}-2\left(w_{4}+w_{1}w_{2}\right)C_{xz}\right\},C_{p2}=\lambda \left(lC_{x}^{2}+w_{3}C_{z}^{2}-w_{4}C_{xz}+w_{1}C_{yx}-w_{2}C_{yz}\right),D_{p2}=1+\lambda \left(lC_{x}^{2}+w_{3}C_{z}^{2}-w_{4}C_{xz}\right)\;\text{and}\;E_{p2}=1+\lambda \left\{\left(w_{1}^{2}+2l\right)C_{x}^{2}+\left(w_{2}^{2}+2w_{3}\right)C_{z}^{2}-2\left(w_{4}+w_{1}w_{2}\right)C_{xz}+2w_{1}C_{yx}-2w_{2}C_{yz}\right\}$$

Therefore, after putting these values the smallest possible *MSE* is given as

(31) $$MSE{\left(ESTp2\right)}_{\min}={\bar{Y}}^{2}\left[1-\frac{A_{p2}D_{p2}^{2}+B_{p2}C_{p2}^{2}-2C_{p2}D_{p2}E_{p2}+B_{p2}+2B_{p2}C_{p2}+D_{p2}^{2}-2D_{p2}D_{p2}}{A_{p2}B_{p2}-E_{p2}^{2}}\right]$$

This Eq. (31) is the second proposed family of estimators for the mean of a finite population under simple random sampling with two auxiliary variables that is deemed efficient under the given conditions for various values of *u, v* and *ℓ.*

## 5 Theoretical comparison

The efficiency of the suggested estimator could be judged through the following conditions in relation to the existing estimators.

### 5.1 For first proposed estimator

Condition (i).

Comparing (1) and (23), MSE(ESTp1)<V(EST0), if

(32) $$\left[\left(\lambda C_{y}^{2}-1\right)+R_{1}\right]>0$$

Where in Eq. (32) $R_{1}=\frac{A_{\mathrm{pr}}D_{\mathrm{pr}}^{2}+B_{\mathrm{pr}}C_{\mathrm{pr}}^{2}-2C_{\mathrm{pr}}D_{\mathrm{pr}}E_{\mathrm{pr}}}{A_{\mathrm{pr}}B_{\mathrm{pr}}-E_{\mathrm{pr}}^{2}}$ and

Condition (ii).

By comparing (3) and (23), MSE(ESTp1)<MSE(ESTr), if Eq. (33) satisfies

(33) $$\left\{\lambda \left(C_{y}^{2}+C_{x}^{2}+C_{z}^{2}-2C_{yx}-2C_{yz}+2C_{xz}\right)-1\right\}+R_{1}>0$$

Condition (iii).

By comparing (5) and (23), MSE(ESTp1)<MSE(ESTrp), if Eq. (34) satisfies

(34) $$\left\{\lambda \left(C_{y}^{2}+C_{x}^{2}+C_{z}^{2}-2C_{yx}+2C_{yz}-2C_{xz}\right)-1\right\}+R_{1}>0$$

Condition (iv).By comparing (7) and (23), MSE(ESTp1)<MSE(ESTreg), if Eq. (35) satisfies

(35) $$\lambda C_{y}^{2}\left(1-\rho_{yx}^{2}-\rho_{yz}^{2}+2\rho_{yx}\rho_{yz}\rho_{xz}\right)-1+R_{1}>0$$

Condition (v).By comparing (9) and (23), MSE(ESTp1)<MSE(ESTs), if Eq. (36) satisfies

(36) $$\left(R_{1}-\frac{\lambda C_{xz}^{2}}{4C_{x}^{2}}-\frac{\Delta_{1}^{2}}{\Delta_{2}}\right)>0$$

Condition (vi).By comparing (11) and (23), MSE(ESTp1)<MSE(ESTh), if Eq. (37) satisfies

(37) $$\lambda C_{y}^{2}\left(1-\rho_{yx}^{2}\right)-H_{1}-H_{2}+R_{1}-1>0$$

Condition (vii).By comparing (13) and (23), MSE(ESTp1)<MSE(ESTsn), if Eq. (38) satisfies

(38) $$R_{1}-R_{3}>0$$

Where $R_{3}=\frac{\Psi_{0}+A_{6}\Psi_{1}+A_{7}\Psi_{2}}{\Psi }$.

Our newly proposed estimator is expected to outperform all other considered estimators under the specified conditions.

### 5.2 For second proposed estimator

The second estimator we introduce in this article is anticipated to exhibit efficiency superior to that of all other estimators, provided the specified conditions are met.

Condition (i).

Comparing (1) and (31), MSE(ESTp2)<V(EST0), if

(39) $$\left[\left(\lambda C_{y}^{2}-1\right)+R_{2}\right]>0$$

Where in Eq. (39) $R_{2}=\frac{A_{p2}B_{p2}^{2}+B_{p2}C_{p2}^{2}-2C_{p2}D_{p2}E_{p2}+B_{p2}+2B_{p2}C_{p2}+D_{p2}^{2}-2D_{p2}E_{p2}}{A_{p2}B_{p2}-E_{p2}^{2}+B_{p2}}$.

Condition (ii).By comparing (3) and (31), MSE(ESTp2)<MSE(ESTr), if Eq. (40) satisfies

(40) $$\left\{\lambda \left(C_{y}^{2}+C_{x}^{2}+C_{z}^{2}-2C_{yx}-2C_{yz}+2C_{xz}\right)-1\right\}+R_{2}>0$$

Condition (iii).

By comparing (5) and (31), MSE(ESTp2)<MSE(ESTrp), if Eq. (41) satisfies

(41) $$\left\{\lambda \left(C_{y}^{2}+C_{x}^{2}+C_{z}^{2}-2C_{yx}+2C_{yz}-2C_{xz}\right)-1\right\}+R_{2}>0$$

Condition (iv).By comparing (7) and (31), MSE(ESTp2)<MSE(ESTreg), if Eq. (42) satisfies

(42) $$\lambda C_{y}^{2}\left(1-\rho_{yx}^{2}-\rho_{yz}^{2}+2\rho_{yx}\rho_{yz}\rho_{xz}\right)-1+R_{2}>0$$

Condition (v).

By comparing (9) and (31), MSE(ESTp2)<MSE(ESTs), if Eq. (43) satisfies

(43) $$\left(R_{2}-\frac{\lambda C_{xz}^{2}}{4C_{x}^{2}}-\frac{\Delta_{1}^{2}}{\Delta_{2}}\right)>0$$

Condition (vi).

By comparing (11) and (31), MSE(ESTp2)<MSE(ESTh), if Eq. (44) satisfies

(44) $$\lambda C_{y}^{2}\left(1-\rho_{yx}^{2}\right)-H_{1}-H_{2}+R_{2}-1>0$$

Condition (vii).

By comparing (13) and (31), MSE(ESTp2)<MSE(ESTsn), if Eq. (45) satisfies

(45) $$R_{2}-R_{3}>0$$

Where $R_{3}=\frac{\Psi_{0}+A_{6}\Psi_{1}+A_{7}\Psi_{2}}{\Psi }$.

Our proposed estimator is expected to surpass all the other estimators, demonstrating superior performance under the conditions specified earlier. Its unique design and methodology position it as a frontrunner in achieving accurate and efficient estimates. This novel approach has a significant impact on the field of estimation.

## 6 Numerical comparison

To evaluate the performance of the suggested estimator on numerical data the below five real world data sets have been considered.

Table 3 shows the MSEs of the existing and proposed estimators for all five datasets given in Table 2. Table 4 presents the PREs of the estimators obtained with respect to the usual estimator of the mean. It is obvious from both tables that in all the above five datasets, the proposed estimators (ESTp1 and ESTp2) surpass all the other estimators; in particular, its efficiency is increased using the transformation. Using different values of the parameters of the auxiliary variables, the efficiency can be further increased.

**Table 2:** Summary statistics of data.

Sr.No	Data	*N*	*n*	$\bar{Y}$	$\bar{X}$	$\bar{Z}$	*C*_*y*_	*C*_*x*_	*C*_*z*_	*ρ*_*yx*_	*ρ*_*yz*_	*ρ*_*xz*_
**1**	[Source: [43]. (District wise tomato production in tones of Pakistan) y: for 2003. x: for 2002. z: for 2001.	97	30	3135.62	3050.28	2743.96	2.206	2.341	2.498	0.81	0.85	0.61
**2**	[Source: [29]. (Area under wheat) Y: in 1974. x: in 1971. z: in 1973.	34	20	856.41	208.88	199.44	0.86	0.72	0.75	0.45	0.45	0.98
**3**	[Source: [1]. y: Number of cultivators, x: Area of the village, z: Number of households in a village.	332	80	1093.1	181.57	143.33	0.763	0.768	0.762	0.97	0.86	0.84
**4**	[Source: [37]. y: Log of leaf burn in second, x: Potassium percentage z: Chlorine percentage.	30	6	0.686	4.654	0.808	0.48	0.23	0.75	0.197	−0.50	0.407
**5**	[Source:[5]. y: Number of "placebo" children, x: Number of paralytic polio cases in the "not in occulted" group, z: Number of paralytic polio cases in the "placebo" group.	34	15	4.92	2.59	2.91	1.012	1.23	1.05	0.73	0.64	0.68

**Table 3:** *MSE*'s of the estimators on real data.

Estimator	Data I	Data II	Data III	Data IV	Data V
EST0	1101857	11168.1	6593.042	0.01447479	0.9241645
ESTr	1367840	26291.25	6755.832	0.08188221	2.009312
ESTrp	2368304	11858.49	7113.921	0.01917153	1.282295
ESTreg	513401.9	11077.64	4764.407	0.009338935	0.6413499
ESTh	159403.1	8795.377	566.1509	0.008119836	0.3907844
ESTs	158074	8794.968	547.6293	0.0299302	0.4150048
ESTsn	75659.99	8824.504	485.232	0.008306754	0.3922845
${\text{ESTp}1}_{1,0}^{1/2}$	11968.63	1599.974	401.5296	0.005866464	0.1002753
${\text{ESTp}1}_{1,C_{z}}^{1/2}$	11902.45	1588.045	397.2231	0.001693495	0.04713765
${\text{ESTp}1}_{\rho ,C_{z}}^{1/2}$	11890.79	1573.642	396.5399	0.007710572	0.03171776
${\text{ESTp}2}_{1,0}^{1/2}$	37996.36	1622.003	407.7981	0.006159058	0.1098727
${\text{ESTp}2}_{1,C_{z}}^{1/2}$	37870.16	1609.83	403.4077	0.001721803	0.05155872
${\text{ESTp}2}_{\rho ,C_{z}}^{1/2}$	37847.94	1595.134	402.7113	0.008225218	0.03491098

**Table 4:** *PRE*'s of the estimators relative to the classical estimator.

Estimator	Data I	Data II	Data III	Data IV	Data V
EST0	100	100	100	100	100
ESTr	80.55453	42.4784	97.59039	17.67757	45.99407
ESTrp	46.52516	94.17817	92.67804	75.50145	72.07115
ESTreg	214.6188	100.8166	138.3812	154.994	144.0968
ESTh	691.2396	126.977	1164.538	178.2645	236.4896
ESTs	697.0516	126.9829	1203.924	48.36181	222.6876
ESTsn	1456.327	126.5579	1358.74	174.2532	235.5853
${\text{ESTp}1}_{1,0}^{1/2}$	9206.209	698.0178	1641.981	246.7378	921.6272
${\text{ESTp}1}_{1,C_{z}}^{1/2}$	9257.397	703.2611	1659.783	854.7286	1960.565
${\text{ESTp}1}_{\rho ,C_{z}}^{1/2}$	9266.473	709.6978	1662.643	187.7265	2913.713
${\text{ESTp}2}_{1,0}^{1/2}$	2899.902	688.5377	1616.742	235.0162	841.1228
${\text{ESTp}2}_{1,C_{z}}^{1/2}$	2909.565	693.7444	1634.337	840.676	1792.45
${\text{ESTp}2}_{\rho ,C_{z}}^{1/2}$	2911.274	700.136	1637.163	175.9806	2647.203

Fig. 1 shows the PREs of the estimators relative to the classical estimator for the population mean, where each line shows the PRE values for different datasets. The graph shows that the PREs are higher for all six estimators (ESTP1(1) to ESTP2(3)) compared with the existing estimators in all datasets. Hence, the suggested families outperform all the other contenders in terms of efficiency when estimating the population mean.

**Fig. 1:** Plotting *PRE*s against each estimator for all populations.

## 7 Simulation study

This section aims at the simulation study of the estimators to check the stability of the estimator in haphazard from sample to sample. Population of size 1000 is taken from multivariate normal distribution for a study variable *y* and two auxiliary variables *X* and *Z*, with mean vector and covariance matrix as

$$\mu =\left[\begin{array}{ccc} 8 & 5 & 6 \end{array}\right]\;\text{and}\;\Sigma =\left[\begin{array}{ccc} 4 & 4 & 5\\ 4 & 9 & 6\\ 5 & 6 & 8 \end{array}\right]$$

where *MSE* and *PRE* values for the existing and proposed estimators were carried out using following steps in R software.

Step-1 Simple random samples without replacement (SRSWOR) of different n = 10, 20, 50, 100, 200. have been drawn from the target population. For each sample size a loop of 10,000 times caried out and allowed R-studio to compute the values of the estimators at each iteration.

Step-2 For each sample, values of the existing and proposed estimators have been carried out separately by taking average of all the iterations.

Step-3 Using values caried out in step-2 the *MSE* of the estimators are obtained.

Step-4 *PRE*s of the estimators are obtained using the following formulae.

$pre\left({EST}_{i}\right)=\frac{Var\left(EST0\right)}{MSE\left({EST}_{i}\right)}\times 100$ where ${EST}_{i}$ replaces different estimators.

Table 5 presents the MSEs of the estimators for all five sample sizes of the simulated data. Table 6 presents the simulation results of the different estimators in simple random sampling with two auxiliaries with respect to the usual estimators for various sample sizes. By exploring the tables, it can be observed that the MSEs of the suggested estimators (ESTp1 and ESTp2) are smaller and the PREs of the suggested families of estimators are higher relative to all the other estimators of the population mean. Further, our estimator is stable with respect to the sample; as the sample size increases, the estimator's efficiency also increases. Therefore, our proposed estimator stands out as the superior choice among the competing estimators under investigation.

**Table 5:** *MSE*s of the estimators for simulation data under different sample sizes.

Estimator	Sample Size (n)				
	10	20	50	100	200
EST0	0.385627	0.195431	0.07506556	0.0352284	0.015755
ESTr	0.2393057	0.111649	0.04167612	0.0194698	0.008718
ESTrp	0.203303	0.101355	0.03856928	0.0182273	0.0082159
ESTreg	0.298997	0.1486294	0.05654175	0.0267619	0.0120430
ESTh	0.292397	0.14714287	0.0563301	0.02635105	0.0117703
ESTs	0.100403	0.05963027	0.01947915	0.0106558	0.004059
ESTsn	0.070037	0.0354237	0.01274426	0.0066930	0.002786
${ESTp1}_{1,0}^{1/2}$	0.021233	0.00815973	0.00262529	0.0012109	0.0005197
${ESTp1}_{1,C_{z}}^{1/2}$	0.019965	0.007396157	0.002485868	0.0010942	0.000475
${ESTp1}_{\rho ,C_{z}}^{1/2}$	0.019533	0.0072857	0.002455432	0.0010255	0.000462
${ESTp2}_{1,0}^{1/2}$	0.0192717	0.0077671	0.00257499	0.0011987	0.0005155
${ESTp2}_{1,C_{z}}^{1/2}$	0.0182076	0.0074235	0.00219178	0.0010217	0.0004517
${ESTp2}_{\rho ,C_{z}}^{1/2}$	0.0178043	0.00720845	0.00208962	0.0010025	0.0004401

**Table 6:** *PRE*s of the estimators with respect to usual estimator for simulated data under different sample sizes.

Estimator	Sample Size (n)				
	10	20	50	100	200
EST0	100	100.00	100.00	100	100.000
ESTr	161.1441	175.0406	180.1165	180.9384	180.719
ESTrp	189.6809	192.8177	194.6253	193.2726	191.7587
ESTreg	128.9734	131.4889	132.7613	131.6362	130.8206
ESTh	131.8846	132.8173	133.2602	133.6888	133.8514
ESTs	384.0781	327.7381	385.3636	330.6024	388.1465
ESTsn	550.605	551.696	589.015	526.347	565.506
${ESTp1}_{1,0}^{1/2}$	1816.168	2395.067	2859.322	3024.929	3031.557
${ESTp1}_{1,C_{z}}^{1/2}$	1931.515	2642.332	3019.692	3219.558	3316.842
${ESTp1}_{\rho ,C_{z}}^{1/2}$	1974.233	2682.392	3057.122	3435.241	3410.173
${ESTp2}_{1,0}^{1/2}$	2000.100	2516.139	2915.183	2938.884	3056.256
${ESTp2}_{1,C_{z}}^{1/2}$	2117.945	2632.599	3424.867	3448.018	3487.934
${ESTp2}_{\rho ,C_{z}}^{1/2}$	2165.921	2711.138	3592.307	3514.055	3579.868

Fig. 2 shows the PREs of the estimators relative to the classical estimator for each sample size for the simulated data. It is obvious from the graph that the PREs for the six proposed estimators (ESTP1(1) to ESTP2(3)) in the simulated data are much higher than those of the existing estimators. Hence, the proposed families are efficient at estimating the population mean among all competitors.

**Fig. 2:** Plotting *PRE*s in different sample size for simulated data.

## 8 Discussion and conclusion

In this study, we introduce two distinct families of exponential-type estimators tailored for application in the context of simple random sampling with dual auxiliary variables. Our analysis extends to the first-order approximation, allowing us to derive expressions for key properties, such as bias and MSE. Notably, we identified the conditions under which our proposed families of estimators outperformed all existing competitors in terms of the MSE.

The effectiveness of these novel families of estimators was further confirmed through rigorous testing of real-world datasets. Our findings consistently revealed lower MSE and higher PRE values compared with all other estimators considered for the same parameter. This underscores the robustness and efficiency of the proposed estimators when applied to practical scenarios.

To ensure the reliability and stability of our estimators across various sample sizes, we conduct extensive simulation studies. Our results, stemming from ten thousand simulations drawn from a tri-variate normal population and spanning five distinct sample sizes (n = 10, n = 20, n = 50, n = 100, n = 200), underscored the efficiency and stability of our proposed estimators under the specified conditions.

In summary, our comprehensive examination of these estimators, supported by both real data analysis and simulation studies, confirms their superiority and efficiency relative to existing competitors in the field. These findings collectively underscore the practical utility of our proposed estimators in simple random sampling with dual auxiliary variables.

## 9 Limitations

Following are some limitations of the proposed estimators.

• These estimators are obtained for the finite populations there is no guarantee that these estimators will be efficient under infinite populations.
• These estimators are designed for only two auxiliary variables scenarios.

## Funding source

The authors received no funding in conducting and processing this research work.

## Data availability statement

The necessary data used in the manuscript are already pre-sent in the manuscript.

## CRediT authorship contribution statement

**Khazan Sher:** Software, Formal analysis, Data curation. **Muhammad Ameeq:** Writing – review & editing, Writing – original draft, Visualization, Validation, Supervision, Software, Resources, Project administration, Methodology, Investigation, Formal analysis, Data curation, Conceptualization. **Muhammad Muneeb Hassan:** Investigation, Funding acquisition, Formal analysis, Data curation, Conceptualization. **Olayan Albalawi:** Data curation, Conceptualization. **Ayesha Afzal:** Validation, Resources, Data curation.

## Declaration of competing interest

The authors declare that they have no known competing financial interests or personal relationships that could have appeared to influence the work reported in this paper.
